# Automatic Segmentation of Calcification Areas in Digital Breast Images

This article has been retracted.

**DOI:** 10.1155/2022/2525433

**Published:** 2022-06-03

**Authors:** Ammar Akram Abdulrazzaq, Yasser Muhammed, Asaad T. Al-Douri, A. A. Hamad Mohamad, Abdelrahman Mohamed Ibrahim

**Affiliations:** ^1^Department of Medical Laboratory Technologies, Al-Maarif University College, Iraq; ^2^College of Technical Engineering, Al-Farahidi University, Baghdad, Iraq; ^3^Department of Dental Industry, College of Medical Technology, Al-Kitab University, Iraq; ^4^Department of Medical Laboratory Techniques, Dijlah University College, Baghdad 10021, Iraq; ^5^The University of Mashreq, Research Center, Baghdad, Iraq; ^6^Accounting and Financial Management, School of Management Studies, University of Khartoum, Sudan

## Abstract

In this study, the authors hope to demonstrate that when mammography is combined with intelligent segmentation techniques, it can become more effective in diagnosing breast abnormalities and aiding in the early detection of breast cancer. In conjunction with intelligent segmentation techniques, mammography can be made more effective in diagnosing breast abnormalities and aiding in the early diagnosis of breast cancer, hence increasing its overall effectiveness. The methodology, which includes some concepts of digital imaging and machine learning techniques, will be described in the following section after a review of the literature on breast cancer (categories, prevention involving the environment and lifestyle, diagnosis, and tracking of the disease) has been completed (neural networks and random forests). It was possible to achieve these results by working with an image collection that previously had questionable regions (per the given technique). Fiji software extracted problematic candidate regions from mammography images, which were subsequently subjected to further examination. To categorize the results of the picture segmentation, they were sorted into three groups, which were as follows: random forest and neural networks both generated promising results in the segmentation of suspicious parts that were emphasized in the highlight of the image, and this was true for both algorithms. Detection of contours of the regions was carried out, indicating that cuts of these segmented sections may be created. Later on, automatic categorization of the targets can be carried out using a learning algorithm, as illustrated in the experiment.

## 1. Introduction

In Arab countries, the large number of women dying from breast cancer makes the disease a significant public health problem, both because of the commotion of morbidity and mortality, as well as the high personal and social cost related to the disease and its treatment, and even more because of the harmful physical and psychological squeal in patients [1]. It is a tumour that originates from breast cells that grow disorderly. 60% to 70% of this type of cancer appears in the form of an “irregular or spheroid” nodule, with speculated, indistinct or microlobulated margins, without calcifications. Close to 20% of cases are nodules with calcifications. Calcifications without an associated nodule constitute just under 20% of all cases [2].

Breast cancer is quite frightening because of its high frequency and the physical (either by total mastectomy or segmental resection – the scar left behind is essential) and psychological (low self-esteem, reduced sexuality, and stigma) that generally harm patients. It is one of the diseases that most cause mortifications and disorders in a wide dimension: it affects the patient, close family members, and caregivers [3].

The most significant risk of this disease is the late diagnosis of the tumour, which can be avoided with digital technologies advancing at an ever-increasing pace to support the early diagnosis of the disease. Mammography, for example, is a test used to diagnose breast abnormalities; it is used in programs for screening women; it reduces the mortality rate due to breast cancer by more than 40% [4], obviously if the diagnosis is still in the preclinical stage, that is, in the early stage of the evolution of malignant tumours.

Because breast cancer is the second with the highest incidence globally and its prevention and mainly treatment are costly for the country's public health, thresholding is a more uncomplicated implementation technique for image processing and computational speed. They are applied very frequently in the image segmentation scenario. It is also called binarization because the technique is based “on partitioning the histogram of the image to convert all pixels [picture element] whose grey tone is greater than or equal to a certain threshold value T into white and the others in blacks” [5].

That said, the question arises: among the many real possibilities of breast cancer prevention, what would be the relevance of the threshold in this effort? The search for answers to this question makes it possible to achieve the objective of this research, which is to discuss the advantages and limits of the threshold technique applied to mammography in the search for areas suspected of malignant neoplastic, facilitating the interpretation of the findings by the physician and, therefore, way, helping the early diagnosis of breast cancer.

### 1.1. Literature Review

Although there is no defined etiology, breast cancer is studied as multifactorial so that certain interacting risk factors determine the disease. Farhadihosseinabadi, et al. (2020) [6] discuss the two categories of risk factors:

1. Modifiable: subject to modifications, interventions, and controls, such as “obesity, high-carbohydrate eating habits, exaggerated consumption of red meat and fats, high intake of alcoholic beverages, the performance of combined hormone replacement therapy for more than five years and excessive radiation exposure” [6]. It is read in Vieira that “overweight is considered a risk factor for the development of the disease and this can be explained by the high estrogen levels resulting from peripheral conversion in adipose tissue”
2. Nonmodifiable: they do not change. They are inherent to the patient, such as gender (higher incidence in females), age (predominance in those over 50 years of age), race, and ethnicity (more frequent among non-Hispanic whites and blacks). Furthermore, the reproductive and hormonal status of women, with early menarche and late menopause one of the most associated, with family history, association when first-degree relatives (mother, sister, daughter, father, brother, and son) developed breast cancer. Mutation in the BRCA1 and BRCA2 genes [7], families carrying these mutations have strong indications for the disease and also the presence of previous breast pathology, women with previous breast cancer have a 1.5x increased risk of developing breast cancer again

How to best prevent breast cancer? This is the question that should be part of the questioning of women, mainly because the answers would allow primary prevention of the disease, that is, before the beginning of the pathological process, even avoiding exposure to many modifiable risk factors, such as the environment and lifestyle, for example, thus preserving health and reducing mortality as a result of this disease.

Some habits should be part of every woman's life, namely, practising physical activities, breastfeeding an infant, regularly eating with fruits, vegetables, fish and nuts, and olive oil, and, on the other hand, avoiding the intake of fat and red meat (which is still not very clear), processed foods, and foods with a high glycemic index, reducing the use of sugar [8].

Therefore, they are simple practices to be cultivated, especially when it is confirmed that, in Arab countries, the risk of having breast cancer is 8% throughout life, which means that one woman in twelve is an expressive risk female. Because of this, the American Society of Mastology, the American Society of Oncological Surgery, and the American Society of Radiology recommend screening the disease in women from the age of forty undergoing mammography annually [4] to detect any breast abnormalities.

Therefore, the early diagnosis of the preclinical stage, even before the presentation of any symptoms, considerably increases the chances of cure. There is secondary prevention, whose main objective is universal and early screening and the performance of mammography, applied “to large populations, in screening programs, significantly reduces mortality rates from breast cancer (reduction above 40%)” [6].

Secondary prevention was aimed at changing the course of the disease since its biological onset has already occurred through interventions that allow its early detection and timely treatment. For this, there must be clear evidence that the disease in question can be identified at an early stage when it is not yet clinically apparent, allowing a practical therapeutic approach, altering its course or minimizing the risks associated with clinical therapy. Furthermore, the resulting drop in morbidity or mortality must be achieved without the adopted strategy's significant burden of adverse effects. Early detection of a disease is possible through education for early diagnosis in symptomatic people or screening (screening) in asymptomatic populations [9].

On the other hand, tertiary prevention occurs in a clinical and symptomatic phase of the disease in the face of findings such as a nodule, oedema—a phase in which mammography is no longer a screening to be diagnostic. “It is important to point out that mammography presents false positives and false negatives, an inherent flaw in the method, but it is the best screening method available at the moment” [10].

There are two groups of mammography exams: screening (in asymptomatic patients, primary prevention, which should be performed annually after age forty in the postmenstrual period) and diagnostic (in symptomatic patients suggestive of breast cancer or even those who need to be supplemented with another exam) [9].

Therefore, early diagnosis and treatment of the disease are essential so that the consequences are less harmful, avoiding or reducing mastectomies and the risk of death. Even if diagnosed early, there are great chances of recovery and even cure. Treatment is usually long, not less than a year. One of the most critical phases is chemotherapy, which, although very effective, its side effects are generally perverse: frequency of nausea, vomiting and mucositis, and somatic changes (alopecia, weight gain, ovarian failure, hormone reduction (testosterone and estrogen causing menopause and vaginal atrophy), various lows, such as libido, vaginal lubrication, anorgasmia, and dyspareunia, affecting sexuality). Inconvenient evaluative judgments emerge for the patient, including the feeling of pity. Even more sinister is the feeling of finitude in the face of the devastating disease [6, 9].

In the face of such nefarious problems, it is never too much to insist on prevention, nor is it too much to insist on good eating and behavioral habits, physical exercise, and a regulated life with sleep patterns, which are basic concepts of public health. We insist that mammography is essential in this prevention, although its sensitivity is approximately 85% and can be reduced to 50% in very dense breasts. In this sense, any alteration identified in the exam must be described according to the Breast Imaging Reporting in the Data System (BI-RADS), “a system created to standardize the reports of breast diagnostic exams regarding the terms used, report creation and recommendation of conduct, which facilitates communication between the multidisciplinary team that assists the patient” [9, 10]. Also, images can be improved using the threshold technique.

## 2. Methodology

It was necessary to obtain a previously classified image bank to evaluate the proposed methodology, with suspicious regions already segmented. [11] provided updated and standardized version of the Digital Database for Screening Mammography (DDSM). The CBIS-DDSM (DDSM Cured Breast Images Subset) dataset includes uncompressed images, data selection, and curation by trained mammographers. In this work, the tool used to extract suspicious candidate regions in mammography images was the Fiji software, a free software distribution of the *ImageJ* project. *Fiji* is a software focused on the analysis of biological images. It relies on the combination of powerful software libraries with a wide variety of scripting languages that allow rapid prototyping of image processing algorithms.

### 2.1. Digital Image

Guzman et al., (2013) [12] define an image as a two-dimensional function *f*(*x*, *y*) of light intensity, where *x* and *y* denote the spatial coordinates of a point and the value of the function *f* (Figure 1) is proportional to the brightness of the image at that point (monochrome image). A digital image is a function *f*(*x*, *y*) discretized in spatial coordinates and brightness. This function produces luminance and reflectance at each point (*x*, *y*).

### 2.2. Monochrome Image

Figure 2, a monochrome image, contains pixels with only one shade of grey (grayscale). Every scale has a minimum and maximum value. In the case of grayscale (with 8 bits), pixels that approach zero are the darkest pixels, while those that approach the maximum value minus one (L-1) are the lightest pixels [13].

### 2.3. Thresholding

It is a technique that separates the regions of an image when it has two classes (the background and the object). Because thresholding produces a binary image as an output, this process is often called binarization. Like the monochromatic image, a binary image is a two-dimensional matrix with only two values. Sometimes they are called logical images: black corresponds to the value 0 and white corresponds to the value 1 [14].

### 2.4. Neural Networks

Neurophysiologist McCulloch and mathematician Walter Pitts in 1943 modelled simple artificial neural networks using electrical circuits. According to McCulloch and Pitts (1943) [15], a neuron can be represented through binary logic (0 or 1). Artificial neural networks emerged from the search to solve problems analogous to the brain (see Figure 3).

### 2.5. Random Forest

Random forest is a classifier that consists of a collection of decision trees. The idea is that if a tree is good, a forest should be even better, as long as there is enough variety within it. The most exciting thing about a random forest is how it creates randomness from a standard dataset.

## 3. Results and Discussion

The segmenting of the candidate suspect regions is based on a feature vector generated for each pixel in the image. In this way, it is possible to obtain a pattern of attributes that can distinguish calcifications. This method uses various image processing filters on the exam image, generating an image of multiple channels. Each image obtained by applying the filters will be used as an attribute for training a machine learning algorithm [16].

As shown in Figures 4 and 5, the machine learning algorithms are provided by the Waikato Environment for Knowledge Analysis (WEKA) data mining and machine learning toolkit [17].

The image filters that best meet the extraction of calcification characteristics in mammographic images were selected through this Fiji plugin.  Figure 6 demonstrates the selection of filters and the learning algorithm used in this study.

Three filters were selected, an edge detector, variance, and maximum value. For each applied filter, new images are generated, making changes to the attributes required for each feature extractor filter. Therefore, the plugin applies different settings for each chosen filter.

In addition to the filter definition settings and the learning algorithm, three classes were defined for the image segmentation result.

Figures 7(a) and 7(b) represent the classes in three colors: red is the sample regions of calcification; the green samples represent other regions of the image; and, finally, purple represents the darkest regions to be ignored.

Once the training samples are defined, the feature vectors will be generated; the values of the sample regions will be used as training data for the random forest algorithm. After the training phase, the prediction will occur for each pixel of the image that will be segmented.

The images resulting from the segmentation algorithm can be seen in Figure 8(a): the first represents the three previously defined classes, and the second is the probability map of the candidate suspect regions.

The algorithm applied for image segmentation returns the probability for each image pixel to belong to the first defined class, calcifications; in this way, Figure 8(b) presents lighter tones for a greater possibility of the suspicious region. The probability of each pixel in the image has a value between 0 (zero) and 1 (one), so 1 (one) corresponds to one hundred percent of accuracy.

To evaluate using the same image feature extraction method, segmentation tests were performed using neural networks as a learning algorithm. The image filters to create the vector of features for each image pixel were the same applied to the random forest algorithm, with only the learning technique being different.

The neural network presented an excellent result in this segmentation methodology. Note that the probability map image presents values closer to white, thus less noise from suspicious regions. The segmentation results, shown in Figures 9(a) and 9(b), demonstrate that it can highlight suspicious regions. Through these probability images, it is possible to detect the contours of the regions; in this way, cuts of these segmented regions can be performed, and, later, an automatic classification of the targets can be performed using a learning algorithm.

## 4. Conclusions

In this study, the relevance of the intelligent segmentation technique associated with the mammography exam in breast cancer diagnosis was evidenced due to the efficiency of image processing and identification of the suspicious region. In this sense, the research's initial objective was to verify that this technique facilitates the interpretation of findings by the physician, greatly helping the early diagnosis of breast cancer.

The results were satisfactory in the test of the segmentation methodology, which seeks to solve problems in a similar way to the human brain, which, in the contour of suspicious segmented regions, made possible cuts and, from which, classify the targets, automatically, with support in a learning algorithm.

The fandom forest algorithm combines several decision criteria to obtain a more accurate prediction, thus allowing more reliable findings, which facilitates physicians' interpretation since suspicious regions are more easily identified.

More studies in this area are needed to improve the technique. Still, it is already possible to dream of a future in which machines and men work together to favor a population, especially when we talk about cancer, a disease whose mortality is still high and little is known about it. Joining forces for early diagnosis is the biggest challenge.

## Figures and Tables

**Figure 1:** Mammography digital image.

**Figure 2:** Monochrome image grayscale.

**Figure 3:** Model of an artificial neuron for collection of decision trees.

**Figure 4:** Banalization for binary image.

**Figure 5:** Model of a random forest.

**Figure 6:** Screen of parameters by segmentation with random forest.

**Figure 7:** (a) Original image. (b) Image with the classes.

**Figure 8:** (a) Prediction using random forest. (b) Random forest probability map.

**Figure 9:** (a) Prediction using neural network. (b) Neural network probability map.

## Data Availability

The data underlying the results presented in the study are available within the manuscript.
